The article "In Vivo Antiplasmodial Potential of the Leaf, Mesocarp, and Epicarp of the Raphia hookeri Plant in Mice Infected with Plasmodium berghei NK65" was published in 2022. Journal: Evid Based Complement Alternat Med.

# In Vivo Antiplasmodial Potential of the Leaf, Mesocarp, and Epicarp of the *Raphia hookeri* Plant in Mice Infected with *Plasmodium berghei* NK65

**DOI:** 10.1155/2022/4129045

**Published:** 2022-07-13

**Authors:** Abimbola Peter Oluyori, Charles Nwonuma, Theresa Akpo, Adejumoke Abosede Inyinbor, Oluwasogo Adewumi Dada, Oluwole Solomon Oladeji, Temitope Aminat Ogunnupebi

**Affiliations:** ^1^Industrial Chemistry Programme, Physical Sciences Department, Landmark University, Omu-Aran, Kwara State, Nigeria; ^2^Landmark University SDG 3: Good Health and Well-Being, Landmark University, PMB 1001, Omu-Aran, Nigeria; ^3^Biochemistry Department, Landmark University, Omu-Aran, Kwara State, Nigeria

## Abstract

**Results:**

The presence of alkaloids, fats and oils, phenolic, and flavonoids was detected via the qualitative test which was confirmed from the result obtained from the GC-MS chromatogram of ethanolic leaves extract. The GC-MS chromatogram of the constituents analogous to the twenty peaks was analyzed as follows: dodecanoic acid (1.94%), 2-undecanone (3.42%), hexadecanoic acid (44.84%), oleic acid (7.45%), octadecanoic acid (8.41%), narcissidine (2.38%), 1-dotriacontanol (2.38%), *α*-sitosterol (2.02%), and lupeol (1.42%). The total phenolics and flavonoids of 118 and 23.3702 mg/g were analyzed in the leaves extract. The leave extract exhibited inhibitory activity of 73.49% against free radicals which could lead to inflammation. The extracts and chloroquine-treated groups showed significant decrease in percentage parasitaemia with pronounced activity observed in chloroquine groups.

**Conclusion:**

The curative and scavenging potencies of studied plant could be attributed to the metabolites analyzed and could guide the formulation of new pharmacophores against malaria infections and inflammations.

## 1. Introduction

Malaria is a disease whose negative impact spans several nations of the world. It is a major health concern in the African continent as different portions of her population are grossly affected. While an estimated 219 million cases of malaria were recorded worldwide in 2017, five countries accounted for about 50% of all the malaria cases with Nigeria contributing 25% of the entire value [1]. A whopping 61% (266,000) of the 435,000 deaths from malaria global deaths recorded in the same year were children under the age of five. All these avoidable deaths may not be unconnected with rising poverty level and illiteracy in the affected countries [2]. Although several successful modern drugs have achieved success in the combat against malaria, there are several concerns. First, the cost of the drug is a major concern for the poor as the means to procure the drug is not there [2–4]. Other reasons include the toxicity of the drug or unpleasant side effects and the emergence of drug-resistant strains of the causative parasite [5–7]. The general belief is that herbs are natural and will provide healing in a more friendly manner. These herbs are sometimes constituted by phytochemicals with novel structures which takes care of drug-resistant malarial parasites. Hence, a continuous search for new antimalarial plants with thorough investigation of the acclaimed antiplasmodial properties is worthy of research attention.

Antimalarial molecules from edible sources may exhibit low toxicological profile and are good candidates for the production of nutraceuticals [8]. An example is the *Raphia hookeri* G. Mann & H. Wendl (*Arecaceae*) fruit which is traditionally recommended for fever infected people in a certain community in Nigeria. This assertion has, however, not been scientifically confirmed. The *Raphia hookeri* palm tree is found commonly in West Africa and is greatly found in the southeastern parts of Nigeria. It is a member of the Palmaceae family which usually grows up to 12 m high. The leaf of this false palm is similar to that of the true palm. However, the fruit is entirely different. Although several studies focused on the nutritional and antioxidant properties of this plant [9], to the best of our knowledge, the antiplasmodial efficacy of the different parts of the plant has not been scientifically authenticated. Hence, this work aimed at the phytochemical investigation and in vivo antiplasmodial activity of the leaf, epicarp, and mesocarp of *R*. *hookeri* plant.

## 2. Materials and Methods

### 2.1. Collection of Plant Materials

*R*. *hookeri* leaf and fruits needed for this study were collected from the premises of Landmark University, Omu-Aran, Kwara State, Nigeria.

### 2.2. Preparation of Extracts

Dried leaf sample (328 g), pulverized epicarp (174.315 g), and mesocarp sample (142.064 g) were macerated in 100 mL of pure ethanol for 5 days at room temperature. The samples were filtered, and the extract solutions were concentrated at a temperature of 60°C using a rotary evaporator. The concentrated extracts were poured into Petri dishes and air-dried before further analysis.

### 2.3. Quantitative Phytochemical Screening

Qualitative phytochemical screening was carried out to identify the presence of flavonoids, phenolics, terpenoids, saponins, and alkaloids in the various plant extracts.

#### 2.3.1. Determination of Total Phenolic Content

To determine the total phenolic contents in the extracts, the Folin–Ciocalteu (FC) method was adopted. In brief, 1 ml of the extract solution was placed in a labelled boiling tube. Afterwards, 1 mL of FC's solution was added followed by 1 mL of 7.5% sodium carbonate solution. After 3 minutes, the mixture was adjusted to 30 mL with deionized water. The mixture was shaken vigorously and allowed to stand for 90 minutes. The absorbance was taken at 765 nm using a UV-visible spectrophotometer, and the total phenolic content was expressed as milligrams per gram gallic acid equivalent [10]. A gallic acid calibration curve was constructed using different concentrations of gallic acid solution (0.02–0.18 mg/ml) (Figure 1). TPC of the plant extracts was determined using the following equation:

(1) $$\begin{array}{c} T=\frac{CxV}{M}, \end{array}$$

where *T* = TPC mg/g GAE, *C* is the concentration of GA established from calibration curve, *V* is the volume of extract in ml, and *M* is the weight of extract in *g*.

#### 2.3.2. Determination of Total Flavonoids

This was done according to a method described by Zhishen et al. [11]. In summary, 1 ml of 2% AlCl_3_ solution in ethanol was added to 1 ml of each extract solution (1 mg/ml). The mixture was shaken vigorously and incubated at room temperature for 15 minutes, after which the absorbance was measured at 430 nm. The total flavonoid content was expressed in mg rutin equivalent (RE)/g extract.

#### 2.3.3. Determination of Total Alkaloids

The total alkaloid content was determined by using a gravimetric method previously described by Obadoni and Ochuko [12]. In brief, a total of 100 mL of 20% acetic acid was added to 1 g each of the dried extracts, taken in a separate 250 mL beaker and covered to stand for 4 h. Each mixture/solution was filtered, and the volume was reduced to one quarter using waterbath. To this sample, concentrated ammonium hydroxide was added drop-wise until the precipitate formation was complete. The whole mixture was allowed to settle, and the precipitate was collected by filtration and weighed to determine the percentage of total alkaloid.

#### 2.3.4. DPPH Radical Scavenging Activity

A method previously described by Ayoola et al. [13] was used to determine the antioxidant potential of the extracts, while ascorbic acid was employed as the standard. Exactly 3 ml of 0.1 mM DPPH solution was placed in a test tube containing 1 ml of the extract solution, and the mixture was incubated in the dark for 30 minutes. The absorbance of the resulting solution was taken at 517 nm. The absorbance of DPPH solution (only) in methanol was also taken at 517 nm using methanol as blank. All determinations were carried out in duplicate and the radical scavenging activity was calculated as follows:

(2) $$\begin{array}{c} \%\text{DPPH scavenging activity}\frac{Ab-Aa}{Ab}x100, \end{array}$$

where *Ab* is the absorption of DPPH in methanol and *Aa* is the absorption of the solution containing the extract.

### 2.4. Antiplasmodial Assays

#### 2.4.1. Animal

A total of 35 Swiss albino mice weighing between 20 and 22 g were used in this study. The animals were obtained from the Institute of Advanced Medical Research and Training (IAMRAT), University Teaching Hospital, Ibadan, Nigeria. The animals were allowed to acclimatize for 8 days preceding the experiments. Animal pellets and water were made available for all the animals. Other handling and care during the study were according to ethical guidelines for handling of laboratory animals. Ethical protocol was approved and issued by the Health Research Ethics of the Biochemistry Department, Landmark University, Nigeria, in line with the international accepted guidelines for laboratory animal use and care.

#### 2.4.2. Parasite

The parasite used in this study was chloroquine-sensitive strain of *Plasmodium berghei* (NK-65 strain) which was obtained from the Institute of Advanced Medical Research and Training (IAMRAT), University Teaching Hospital, Ibadan, Nigeria.

#### 2.4.3. Grouping and Malaria Parasite Inoculation

The experimental mice were grouped into five (3 mice) and housed in plastic cages with frequent monitoring and feeding. Group 1 mice were treated with 8 mg/kg chloroquine (positive control), group 2 were treated with epicarp extract of *R*. *hookeri*, group 3 with mesocarp extract, group 4 with endocarp extract, while group 5 received no treatment (negative control). The experimental mice were inoculated by intraperitoneal injection with standard inoculum of *Plasmodium berghei*. The infected mice were left for four days in order to allow the parasite to establish.

#### 2.4.4. Determination of Parasitaemia

Curative effects of ethanolic extracts from different parts of *R. hookeri* plant were investigated using the curative test. On day 4 (postinoculation), about 0.2 ml of 200 mg/kg and 8 mg/kg of the extracts and chloroquine (CQ), respectively, were administered, while group 5 received no treatment. The administration was carried out once in 24 h for 8 days. Blood smear from each group was obtained from the mice tails on day 4, 7, 9, and 11. These blood samples were smeared on microscope slides to make both the thick and thin film. The blood films were fixed in 100% methanol and then stained with Giemsa prepared with buffered water (pH 7.2). Parasitaemia was examined microscopically (using *x* 100 immersion oil objective). Percentage parasitaemia and inhibition were calculated according to the following equations.

(3) $$\begin{array}{c} \text{Average}\%\text{parasitaemia}=\frac{\text{Number of parasitized erythrocytes}}{\text{Total number of erythrocytes}}X100\%,\\ \%\text{inhibition}=\frac{\%\text{parasitaemia control}-\%\text{parasitaemia}-\text{treated group}}{\%\text{parasitaemia in the control group}}X100\%. \end{array}$$

#### 2.4.5. Determination of Packed Cell Volume (PCV)

The packed cell volume (PCV) of the groups was recorded to monitor any variation that could occur during the course of infection and treatment. Blood sample was taken from each control and extract groups on day 11 to compare the effects on erythrocytes level in blood serum of the mice. The PCV values were then calculated according to the method of Endale et al. [14].

(4) $$\begin{array}{c} \text{PCV}=\frac{\text{Volume of erythrocytes in given blood X }100}{\text{Total blood volume}}. \end{array}$$

### 2.5. GC-MS Analysis

The identification of bioactive secondary metabolites present in leaf extract of *R*. *hookeri* was determined by GC-MS (Agilent 7890 A) with the following parameters: injection temperature: 270°C and detector temperature: 320^o^C. The first step of this GC program was at 40°C for two minutes; ramp from 10°C/minute to 310°C at 16 minutes. The injection volume for all the samples was 1 *μ*L, and the National Institute of Standard and Technology (NIST) library database was used to interpret the mass spectrum.

### 2.6. Statistical Analysis

Two-way ANOVA (with Bonferroni posttest) was used to analyze the antiplasmodial data using GraphPad Prism 5 software.

## 3. Results

### 3.1. Qualitative Phytochemical Screening

The qualitative assessment of secondary metabolites in the mesocarp, leaf, and epicarp of *R*. *hookeri* showed the presence of some important compounds (Table 1).

All the extracts with the exception of the leaf had notable presence of fats and oil as well as alkaloids, while only the leaf was exceptionally rich in flavonoids and phenolics. However, none of the extracts tested positive to the saponins' froth test. Hence, the quantitative presence of alkaloids, phenolics, and flavonoids was subsequently investigated.

### 3.2. Quantitative Phytochemical Investigation

#### 3.2.1. Total Phenolic Content

The total phenolic content (TPC) of the epicarp, mesocarp, endocarp, and leaf extracts were estimated using the Folin–Ciocalteu method and the results were expressed in mg/g of the crude extracts. According to Table 2, TPC of the extracts investigated ranges from 10.11 to 117.00 mg/g GAE. The highest concentration of TPC was observed in the leaf (117.00 mg/g GAE), followed by the epicarp (54.60 mg/g GAE); while, the mesocarp (10.11 mg/g GAE) had the lowest phenolic concentration.

### 3.3. Total Flavonoid Content

The total flavonoid content of the crude extracts of *R*. *hookeri* was evaluated from the Rutin calibration curve and expressed as mg RE/g of dry materials.

The highest flavonoid content was displayed by ethanolic extracts of leaf with concentration of 23.3702 mg/g RE; while, the mesocarp showed the lowest concentration of 0.4942 mg/g RE (Table 3).

### 3.4. Total Alkaloid Content

The gravimetric analysis for total alkaloid contents in the investigated part of *R*. *hookeri* showed that high alkaloid contents were present in the epicarp (29.4 mg/1.00 g of sample), followed by the mesocarp (17.6 mg/1.00 g); while, the leaf had the least alkaloid contents (15.9 mg/1.00 g of sample).

### 3.5. DPPH Radical Scavenging Activity

The DPPH (1,1-diphenyl-2-picrylhydrazyl radical) assay, which is the most common technique in the determination of antioxidant activity of plant-derived from molecules, was employed in this study. Once the DPPH encounters free radical scavengers, the purple colour rapidly fades away. In this research, the radical scavenging activity of the different parts of *R*. *hookeri* plants was evaluated using ascorbic acid as a standard at different concentrations. The results showed that the leaf had the highest antioxidant activity followed by the epicarp (Figure 1).

### 3.6. In Vivo Antimalarial Assay of Crude Extracts

#### 3.6.1. Effects of the Extracts on Packed Cell Volume (PCV)

The effects of crude extracts of *R*. *hookeri*, CQ, and controls were investigated in the experimental mice before inoculation with *Plasmodium* strain (NK65) and after inoculation. According to Figure 2, there is a significant reduction in the level of blood erythrocytes after treatment, with the lowest PCV observed in the mesocarp-treated group. CQ and leaf extract exhibited similar results, while mesocarp exhibited close effects on blood serum (erythrocytic level).

#### 3.6.2. Effects of the Extracts on Level of Parasitaemia

The extracts and CQ-treated groups showed a significant decrease in percentage parasitaemia with pronounced observed in CQ groups. While CQ significantly inhibited the growth of *Plasmodium* in infected mice after post-eight-day treatment showing inhibitory activity of 100% (Table 4), the activity observed in the leaf extract was encouraging with % inhibition ranging from −16.51 to 74.21% after oral administration of the extract for 8 days.

The mesocarp exhibited the lowest inhibitory activity (67.76%) when compared with epicarp (71.20%) and leaf extract (74.21%).

### 3.7. GC-MS Analysis of *R*. *hookeri* Leaf

GC-MS analysis of crude extract of *R*. *hookeri* leaf revealed the presence of some important phytochemicals (Figure 3) such as phenols, terpenoids, alcohols, sterols, organic aliphatic, and esters (Table 5).

The GC-MS chromatogram of the constituents analogous to the twenty peaks was analyzed as follows: dodecanoic acid (1.94%), 2-undecanone (3.42%), hexadecanoic acid (44.84%), hexadecanoic acid, ethyl ester (3.50%), oleic acid (7.45%), octadecanoic acid (8.41%), narcissidine (2.38%), 1-dotriacontanol (2.38%), *α*-sitosterol (2.02%), and lupeol (1.42%). The libraries of identified secondary metabolites are shown in Figure 4. Among these, hexadecanoic acid had the highest percentage composition (44.84%), while the least abundant compound is lupeol (1.42%).

## 4. Discussion

Generally, phytochemicals play significant roles in plants and the reported therapeutic efficacies could be linked to these compounds. Medicinal plants since time immemorial have standout as effective curative agents in ameliorating diseases or infections. The ethnobotanical and ethnopharmacological studies of plants could be connected to several secondary metabolites or pharmacophores isolated from plants. According to scientific reports, several pharmacophores or metabolites have exhibited strong inhibitory activity against different pathogenic or parasitic infections such as malaria, cholera, typhoid, and tuberculosis [4, 28]. Phenolics, flavonoids, alkaloids, fats, and oils were among the phytochemicals detected by the qualitative tests. However, contrary to an earlier observation [9], the saponins in the epicarp and the leaf extract were below the detectable level as none of the extracts tested positive to the saponins froth test. Hence, further research is required in this direction.

The PCV of the treated and untreated groups were studied before inoculation, after inoculation, and during treatment. A significant reduction was observed in the PCV of infected mice which could be linked to one of the symptoms of malaria infection. The loss in PCV could also be linked to the spread or growth of *Plasmodium* infections in the studied organisms. From observation, a significant increase in PCV after treatment with different dosage of extracts could be associated to curative potentials of the extracts. The feed compositions are known to contain high calories, carbohydrates, mineral salts, and vitamins which are required for proper growth and development of organisms. The variations in PCV could be associated with dose concentrations and polarity of the extracts with polar extracts showing a significant increase [29, 30].

In folk medicine, different parts of *R. hookeri* are widely used for the treatment of parasitic infections such as malaria, diabetes, and cholera [31–33]. Generally, symptoms such as body pains, fever, weight loss, low erythrocytes, and headache could be linked to malarial infection. These symptoms are common in people in tropical or subtropical regions, especially those close to the equator. It is well noted that decoction or infusion from plants could function as analgesic, antipyretic, or immune stimulating therapies that could give characteristic relief. Some secondary metabolites such as terpenoids, alkaloids, rutin, and gallic acid have significantly reduced parasitaemia level in experimental mice; however, these metabolites may not be enough to fully elucidate the total effects of plant extracts [34, 35]. Furthermore, the observed parasitaemia curative potential of the extracts in the treated groups may be attributed to the presence of various secondary metabolites such as alkaloids and phenolics analyzed [9]. Specifically, the phenolics are likely to be responsible for the antiparasitic activity, since the leaf, which showed the highest phenolic content, also displayed the strongest parasitaemia inhibition (curative potential). Furthermore, the PCV of all groups of treated mice improved, as shown in Figure 2.

This study also validated the application of GC-MS as an indispensable analytical technique for the identification of bioresource or secondary metabolites in plant materials. The analysis of the ethanol extract of *R. hookeri* leaves revealed the presence of 20 bioactive metabolites. Amongst the analyzed metabolites, the presence of fatty acids such as dodecanoic acid, tetradecanoic acid, hexadecanoic acid, hexadecanoic acid ethyl ester, oleic acid, octadecanoic acid, and octadecanoic acid ethyl ester could be linked to the pronounced antioxidant activity exhibited by leaf extract of this plant [36, 37]. Several studies have reported high biological activity of leaf extracts [9, 38]. The reported pharmacological activity of leaves extracts could be due to variety of bioactive metabolites present because it is an important part of the plant which aids in absorbing food, water, and air from sunlight and atmosphere.

To the best of our knowledge, reports on the bioactive constituents of *R. hookeri* leaves, epicarp, and mesocarp extracts are scarce, and this is the first report about their antiplasmodial potential. Particularly, the ethanolic extract of leaves of *R. hookeri* contains an array of phytochemicals which could be processed into plant-based pharmaceuticals or drugs for the treatment of malaria, microbial infections, inflammation, cancer, and infertility.

## 5. Conclusion

The current result using GC-MS analysis of leaves of *R. hookeri* showed that it contains some essential bioactive secondary metabolites. These metabolites could be linked to the marked antiplasmodial and antioxidant activities exhibited by leaves, epicarp, and mesocarp extracts of the plant. Although the parasite was not totally cleared, the leaf extract exhibited an impressive parasitaemia suppression which is worthy of further investigation. The pronounced inhibitory activities against *Plasmodium* species suggested that different parts of *R. hookeri* plant could be applicable in the treatment of malaria and scavenge free radicals and reactive oxygen species that contribute to several human ailments. The results suggest that secondary metabolites analyzed from studied plants may warrant further investigation which could lead to the isolation of novel phytochemicals and improved therapeutic applications.

## Figures and Tables

**Figure 1:** DPPH radical scavenging activity of different parts of the *R*. *hookeri* plant.

**Figure 2:** PCV of extracts and control-treated experimental groups.

**Figure 3:** GC-MS chromatogram of crude extract of *R*. *hookeri*.

**Figure 4:** Structural moiety of selected compounds from GC-MS of *R*. *hookeri* leaf extract.

**Table 1:** Qualitative phytochemical screening of *R*. *hookeri* ethanolic extracts.

S/N	Test	Mesocarp	Leaf	Epicarp
1	Flavonoids	−	+	−
2	Alkaloids	+	−	+
3	Fat and oils	++	_	+
4	Saponins	−	−	−
5	Phenolics	−	_+_	−

**Table 2:** Total phenolic content of *R*. *hookeri* extracts.

S/N	Extract	Total phenolic (mg GAE/g)
1	Leaf	117.00
2	Epicarp	54.60
3	Mesocarp	10.11

**Table 3:** Total flavonoid content of *R*. *hookeri* extracts.

Extract	Total flavonoid content (mg/g RE)
Mesocarp	0.494234
Leaf	23.3702
Epicarp	0.964933

**Table 4:** The percentage parasitaemia and inhibition of the extracts and chloroquine on the level of parasitaemia in experimental mice after post-four-day treatment (D8) (*n* = 2).

Drug/dose mg/kg		Day 4	Day 7	Day 9	Day 11
Control	% parasitaemia	2.06 ± 0.23^a^	5.25 ± 2.55^a^	14.53 ± 3.98^a^	62.46 ± 7.55^a^
	% inhibition	0	0	0	0

Chloroquine	% parasitaemia	2.28 ± 0.20^a^	0.00 ± 0.00^a^	0.00 ± 0.00^a^	0.00 ± 0.00^b^
	% cure	−10.68	100	100	100

Mesocarp extract	% parasitaemia	0.71 ± 0.405^a^	2.73 ± 0.315^a^	16.63 ± 5.930^a.c^	20.14 ± 0.820^a,c^
	% inhibition	65.78	48.1	−14.45	67.76

Epicarp extract	% parasitaemia	3.00 ± 0.775^a^	13.19 ± 6.99^a^	13.92 ± 1.87^a^	17.99 ± 8.17^a,c^
	% inhibition	−45.63	−151.24	4.2	71.2

Leaf extract	% parasitaemia	2.40 ± 1.93^a^	3.38 ± 0.90^a^	7.02 ± 3.49^a^	16.11 ± 13.68^a,c^
	% inhibition	−16.51	35.62	51.69	74.21

Each value represents mean ± SEM (standard error of the mean). Values with different letters are significantly different at (*p* < 0.05).

**Table 5:** The phytochemicals detected in the crude extract of *R*. *hookeri* leaf.

Peak	Retention time	Area (%)	Phytoconstituents	Molecular formula (weight)	Biological activity
1	9.845	1.94	Dodecanoic acid (fatty acid)	C_12_H_24_O_2_ (200.318)	Antiviral and antibacterial [15]
2	11.086	2.13	Tetradecanoic acid (fatty acid)	C_14_H_28_O_2_ (228.370)	Antibacterial and antioxidant [16]
3	11.557	1.49	Oley alcohol (unsaturated fatty alcohol)	C_18_H_36_O (268.478)	Antimicrobial [17]
4	11.598	3.42	2-Undecanone (dialkyl ketone)	CH_3_(CH_2_)_8_COCH_3_ (170.290)	Antimicrobial and antioxidant [18]
5	12.263	44.84	Hexadecanoic acid (fatty acid)	C_16_H_32_O_2_ (256.400)	Antibacterial [19]
6	12.410	3.50	Hexadecanoic acid, ethyl ester (fatty acid)	C_18_H_36_O_2_ (284.500)	Antibacterial [19]
7	13.174	3.40	Phytol (diterpene alcohol)	C_20_H_40_O (296.530)	Antimicrobial [20]
8	13.339	7.45	Oleic acid (fatty acid)	C_18_H_34_O_2_ (282.47)	Antifungal [21]
9	13.480	8.41	Octadecanoic acid (fatty acid)	C_18_H_36_O_2_ (284.480)	Antibacterial [22]
10	13.692	1.73	Octadecanoic acid ethyl ester (fatty acid)	C_20_H_40_O (312.530)	Antibacterial [22]
11	15.180	2.41	4,8,12,16-Tetramethylheptadecan-4-olide (fatty acid)	C_21_H_40_O_2_ (324.541)	Antidepressant [23]
12	16.986	3.68	Hexadecanoic acid, 2-hydroxy-1-(hydroxymethyl) ethyl ester (fatty acid)	C_19_H_38_O (330.503)	Antimicrobial [24]
13	20.756	1.86	Octadecanoic acid, 2-hydroxy-1-(hydroxymethyl) ethyl ester (fatty acid)	C_21_H_42_O (358.556)	Antimicrobial [25]
14	23.050	2.38	Narcissidine (alkaloids)	C_18_H_23_NO_5_ (333.400)	Antimicrobial [26]
15	23.356	2.94	4,7-Dimethyl-5-decyne,4,7-diol (alcohol)	C_12_H_22_O_2_ (198.302)	Antioxidant [27]
16	23.591	1.56	1-Dotriacontanol (alcohol)	C_32_H_66_O (466.870)	
17	23.903	1.50	2-Heptacosanone	C_27_H_54_O (394.700)	Antimicrobial [25]
18	27.168	1.93	1-Eicosanol (alcohol)	C_20_H_42_O (298.555)	Antibacterial [24]
19	32.544	2.02	*α*-Sitosterol (phytosterols)	C_29_H_50_O (414.710)	Antimicrobial [25]
20	34.920	1.42	Lupeol (pentacyclic triterpenoids)	C_30_H_50_O (426.720)	Antimicrobial [25]

## Data Availability

The data used to support the findings of this study are available from the corresponding author upon request.
